# Improving Node Classification through Convolutional Networks Built on Enhanced Message-Passing Graph

**DOI:** 10.1155/2022/3999144

**Published:** 2022-09-23

**Authors:** Yu Song, Shan Lu, Dehong Qiu

**Affiliations:** School of Software Engineering, Huazhong University of Science and Technology, Wuhan 430074, China

## Abstract

Enhancing message propagation is critical for solving the problem of node classification in sparse graph with few labels. The recently popularized Graph Convolutional Network (GCN) lacks the ability to propagate messages effectively to distant nodes because of over-smoothing. Besides, the GCN with numerous trainable parameters suffers from overfitting when the labeled nodes are scarce. This article addresses the problem via building GCN on Enhanced Message-Passing Graph (EMPG). The key idea is that node classification can benefit from various variants of the input graph that can propagate messages more efficiently, based on the assumption that the structure of each variant is reasonable when more unlabeled nodes are labeled properly. Specifically, the proposed method first maps the nodes to a latent space through graph embedding that captures the structural information of the input graph. Considering the node attributes together, the proposed method constructs the EMPG by adding connections between the nodes in close proximity in the latent space. With the help of the added connections, the EMPG allows a node to propagate its message to the right nodes at long distances, so that the GCN built on the EMPG need not stack multiple layers. As a result, over-smoothing is avoided. However, dense connections may cause message propagation saturation and lead to overfitting. Seeing the EMPG as an accumulation of some potential variants of the original graph, the proposed method utilizes dropout to extract a group of variants from the EMPG and then builds multichannel GCNs on them. The multichannel features learned from different dropout EMPGs are aggregated to compute the final prediction jointly. The proposed method is flexible, as a brod range of GCNs can be incorporated easily. Additionally, it is efficient and robust. Experimental results demonstrate that the proposed method yields improvements in node classification.

## 1. Introduction

Graphs are a pervasive data structure in different disciplines. A problem that comes up often but has remained largely unaddressed is node classification, especially when the graphs are sparse and with few labels. The aim of node classification is to infer the category of the unlabeled nodes by using the given labeled nodes and the graph structure. A large number of methods for semi-supervised node classification have been proposed. The earlier work was done by using structural information only [1–6]. Recently, attention has shifted to Graph Convolutional Networks (GCNs) [7–14]. The GCNs model graph structure and node attribute jointly, and have been very promising.

Most GCNs work by a message-passing scheme. A Graph Convolutional Layer (GCL) can be viewed as a message-passing step. In a layer, each node sends its feature representation, i.e., the “message,” to its neighbors, and then updates its feature representation by aggregating all “messages” received from its neighbors. Different aggregation and update functions lead to different GCNs, which yield different results. Due to this flexibility, the class of message-passing networks has been widely used in various applications, including but not limited to publication citation networks [7–12], social networks [15], applied chemistry [16], natural language processing [17], and brain-computer interface [18], and have recently achieved great success.

Despite the fruitful progress, the limitation of GCNs has also been revealed as the study of GCN advances. For example, the first GCN [7], which updates node features by aggregating messages from one-hop neighbors, lacks the ability to receive long-range messages. This suggests it only works on the graphs where the nodes from the same class tend to be connected directly. However, in many practical graph data, the nodes with the same label may be far apart from each other in the graph, even though they possess high structural similarity. That is, the graphs do not or only partly satisfy the homophily assumption [19]. As shown by the toy example plotted in the upper left corner of Figure 1, the articles on the same topic but published by independent research groups may be separated in the citation network, where the node color represents the article label. In cases like this, the performance of the GCNs that do not have the means to capture long-range messages drops quickly, especially where the labeled nodes are scarce and the graph is sparse [20, 21]. It is therefore important to enhance message propagation to realize information exchange between long-distance nodes.

However, there are significant challenges facing researchers when addressing the problem. One straightforward way to expand message propagation is to stack more layers to build deep GCNs. Theoretically, a *k*-layer network can propagate messages from a node to the nodes at *k*-hop distance. Unfortunately, stacking more layers tends to cause the problem called over-smoothing [22], because repeatedly applying Laplacian smoothing in a deep network would mix the node features and make them indistinguishable. Besides, deep networks may cause over-crashing [23]. Furthermore, deep networks are more difficult to train.

Another way to enhance message propagation is to add connections. To mitigate over-smoothing in deep networks, some researchers introduced jumping connections or dense connections to realize multi-hop message propagation [24, 25]. On the other hand, some researchers attempted to combine dense connections with shallow GCNs [8, 13, 26–28]. However, too dense connections not only make learning model complex, but also cause the problem of overfitting, especially when the labeled nodes are scarce [29, 30]. Additionally, as will be discussed in this article, too dense connections cause message propagation saturation and bring noise in message propagation, which would certainly decrease the accuracy of node classification.

This article proposes a new method to cope with the challenges. The proposed method first generates Enhanced Message-Passing Graph (EMPG) and then builds multi-channel GCNs on different dropout EMPGs, such that the long-distance messages can be aggregated in an effective way by shallow GCNs and the impact of label scarcity and graph sparsity can be mitigated simultaneously. Unlike the jumping connections that are added into deep GCNs to link the output of low layers to the input of high layers [24, 27], the connections are added between the nodes that are similar in terms of structural proximity in a latent space where the graph is embedded. This operation is reasonable, because the nodes with similar labels have a larger probability of being neighbors [31, 32]. These added connections allow propagating messages between long-range nodes without the need of increasing convolutional layers. Thus, the problem of over-smoothing is avoided.

Meanwhile, the multi-channel GCNs built on different dropout EMPGs well combat the problem of overfitting caused by label scarcity and too dense connections. Various techniques have been developed to tackle overfitting, an incomplete list includes early stopping [33, 34], data augmentation [35, 36], adding statistical noise to inputs [37], and regularization [38–40]. Dropout, which was first introduced by Hinton et al. [41] and subsequently proved to be a stochastic regularization technique by Srivastava et al. [42], is an effective technique for tackling overfitting. Dropout can be applied to nodes [15] or edges [43]. Because it is reasonable to view the EMPG as an accumulation of some potential variants of the input graph, we apply dropout to the EMPG instead of to the input graph. A series of variants of the input graph is extracted by dropping EMPG edges out randomly, which is equivalent to augmenting the input data. Besides, dropping EMPG edges out randomly can prevent message propagation saturation and reduce noise.

The scheme of adding connections and the way of employing the added connections proposed in this article are different from the existing work [12, 26, 28]. Furthermore, our method adopts a multi-channel aggregation architecture that is different from the two-channel architecture [12] and the bi-level aggregation architecture [28]. Multi-channel neural networks are effective at combining information from different views [44, 45]. The difference between the proposed method and the existing work will be compared and discussed in detail in the relevant section of this article. The results of extensive experiments on benchmark datasets show that the proposed method outperforms the baseline methods on the task of node classification in terms of classification accuracy. We summarize the contributions of this article as follows:

1. A dense connection scheme based on graph embedding is proposed for enhancing message propagation over long-range nodes in GCNs without the need of increasing convolutional layers, which therefore can prevent over-smoothing.
2. A multi-channel GCN architecture is constructed to learn node representation from a group of variants of the input graph. The architecture leverages the strengths of the augmented training data that possess the same underlying distribution of the input graph and keeps the complexity of the GCN in each channel low, so that it can avoid overfitting.
3. The experimental results demonstrate the superiority of the proposed method in contrast with other state-of-the-art methods on the task of node classification in sparse graph with few labels.

The rest of this aticle is organized as follows.  Section 2 presents the motivation and the method framework.  Section 3 describes the method implementation in detail. In Section 4, extensive experiments on benchmark datasets are conducted to evaluate the proposed method. A review of related work is provided in Section 5. Finally, Section 6 concludes this article and presents future work.

## 2. Motivation and Method Framework

In this section, we present the motivation after introducing relevant background knowledge and then put forward the method framework.

### 2.1. Motivation

Let *𝒢*=(*𝒱*, *ℰ*) be an undirected graph with a node set *𝒱* and an edge set *ℰ*. *N*=|*V*| is the number of nodes and *M*=|*E*| is the number of edges. The weight of the edge (*v*_*i*_, *v*_*j*_) ∈ *E* is stored by the element *a*_*ij*_ of the adjacency matrix *A* ∈ *R*^*N*×*N*^. The node features are denoted by *X*={*x*_1_, ⋯, *x*_N_} ∈ *ℝ*^*N*×*d*^, where *x*_*i*_ ∈ *ℝ*^*d*^ is the feature vector of the node *v*_*i*_ ∈ *V*. *Y* ∈ {0,1}^*N*×*C*^ is the label matrix, where *C* is the number of node categories. The node set *𝒱* is divided into a labeled node set *𝒱*_L_ and an unlabeled node set *𝒱*_U_. In this article, we address the problem of semi-supervised node classification over sparse graph with few labels, that is, |*ℰ*| ≪ |*𝒱*|^2^ and |*𝒱*_L_| ≪ |*𝒱*|. Our goal is to build a classifier *f*_A,X,Y,v_i_∈*𝒱*_U__(v_i_)⟶y that predicts the label of the nodes of *𝒱*_U_ based on the adjacency matrix A, the node feature matrix X, and the label matrix Y.

The GCN developed by Kipf and Welling [7] achieved great success in semi-supervised node classification. The feed-forward propagation in GCN is recursively conducted as follows:

(1) $$\begin{array}{c} H^{\left(k+1\right)}=ReLU\left(\hat{A}H^{\left(k\right)}W^{\left(k\right)}\right)\text{,} \end{array}$$

where *H*^(*k*)^={*h*_1_^(*k*)^, ⋯, *h*_*N*_^(*k*)^} are the hidden vectors of the *k*-th layer with *h*_*i*_^(*k*)^ as the hidden feature for the node *v*_*i*_; $\hat{A}={\hat{D}}^{-1/2}\left(A+I\right){\hat{D}}^{-1/2}$ is the re-normalization of the adjacency matrix A and $\hat{D}$ is the corresponding degree matrix of (A+I); W^(k)^ ∈ *ℝ*^*D*^(*k*)^×*D*^(*k* − 1)^^ is the filter matrix of the *k*-th layer and *D*^(*k*)^ is the size of the *k*-th layer.

Soon afterward different variants of GCN emerged. Most of them focus on improving message propagation and aggregation across network. For example, Wu et al. [8] proposed an efficient network name SGC by removing the nonlinearities between layers:

(2) $$\begin{array}{c} H={\hat{A}}^{k}XW^{\left(0\right)}W^{\left(1\right)}\cdots W^{\left(k\right)}={\hat{A}}^{k}X\tilde{W}={\hat{S}}^{k}\tilde{W,} \end{array}$$

where ${\hat{S}}^{k}={\hat{A}}^{k}X$ is a feature extraction/smoothing component. Xu et al. [24] combined all previous representations [*H*^(1)^, ⋯, *H*^(k)^] to learn the final representation. Li et al. [25] incorporated residual layers, dense connections, and dilated convolutions into GCN architecture. APPNP [46] adopts *k*-hop aggregation. Sun et al. [47] combined the predictions from different orders of neighbors by using AdaBoost.

We abstract the GCN and its variants into a block diagram shown in Figure 2, which depicts the general organization and the recursive training process. It can be found that the main difference between the GCNs mentioned above lies in the way of using the representations *H*^(1)^, ⋯, *H*^(*k*)^ of all intermediate layers to learn the final representation. The existing models focus either on increasing the number of layers *k*, or on finding a particular way to combine *H*^(1)^, ⋯, *H*^(*k*)^. However, with the increase of convolutional layers, the output features may be over-smoothed and converge to the same values. Additionally, stacking more layers into a GCN increases its complexity and makes it much more difficult to train. What is worse, a complex model with numerous trainable parameters easily tends to overfit training samples, especially when training samples are scarce.

To overcome the weaknesses, we put effort into modifying the block $\hat{A}$ to improve its efficiency in message propagation. As shown in Figure 2, the block $\hat{A}$ plays an important role in model learning. By modifying $\hat{A}$, a model can propagate messages efficiently from a node to the appropriate nodes at long distances. Enhancing message propagation is critical for semi-supervised node classification, especially when the labeled nodes are scarce. In the original GCN proposed by Kipf and Welling [7], $\hat{A}={\hat{D}}^{-1/2}\left(A+I\right){\hat{D}}^{-1/2}$ is generated from the graph with a self-loop attached to each node. The attached self-loops could be regarded as a special way of enhancing node messages. In the next section, we present a new dense connection scheme for enhancing message propagation over long-range nodes.

### 2.2. Method Framework

Motivated by the above discussion, we propose the framework of our method as shown in Figure 1. The most important step is to generate the EMPG that enhances message propagation efficiently. To this end, we first map the input graph *𝒢*=(*𝒱*, *ℰ*) to a continuous latent space, and then construct the EMPG *𝒢*′=(*𝒱*, *ℰ*′) by adding connections between the nodes that are structurally similar. Because the EMPG allows nodes to propagate messages to the right nodes that are far apart in the input graph, it is not needed to stack many layers into a GCN to realize long-range message propagation. However, the EMPG is too densely connected. A reasonable understanding of the EMPG is to view it as an accumulation of some potential variants of the input graph. Therefore, the next step is to generate a group of dropout EMPGs by removing some edges from the EMPG randomly. Each dropout EMPG *𝒢*_drop_′=(*𝒱*, *ℰ*_drop_′) works as a substitute for the input graph *𝒢*=(*𝒱*, *ℰ*) to train a GCN. This is equivalent to augmenting the input data. As a result, the potential risk of overfitting is reduced. Additionally, by removing edges from the EMPG *𝒢*′=(*𝒱*, *ℰ*′) randomly, we can avoid message propagation saturation and mitigate noise, the two most common adverse effects caused by the added connections. Finally, we train the multi-channel GCNs built on different dropout EMPG *𝒢*_dr op_′=(*𝒱*, *ℰ*_dr op_′) and combine the multi-channel outputs together to produce the final prediction.

## 3. Method Implementation

In this section, we describe the proposed method in detail, focusing on two main parts: (i) generating EMPG based on graph embedding and (ii) constructing multi-channel GCNs on dropout EMPGs.

### 3.1. Generating EMPG Based on Graph Embedding

#### 3.1.1. Graph Embedding

Graph embedding is vital to EMPG generation. Given the input graph *𝒢*=(*𝒱*, *ℰ*), graph embedding maps each node v ∈ *𝒱* to a vector *z*_*v*_ ∈ *ℝ*^*d*^, where *d* is the dimensionality of the latent space. It is required that graph embedding preserves the graph structure effectively. There are several methods that can embed a graph into a latent Euclidean space according to the graph structure [48–50]. Among them, DeepWalk [48] relies on truncated random walk and uses a skip-gram model to generate node embeddings. Since DeepWalk can preserve the local structure around each node well, it is chosen to map the input graph *𝒢*=(*𝒱*, *ℰ*). Certainly, other suitable graph embedding methods could be used for different applications.

#### 3.1.2. Adding Connections

The next step extracts the structural neighborhood for each node v ∈ *𝒱*, using the result of graph embedding. The structural neighborhood of the node v, denoted by *𝒩*_z_(v), contains the nodes that are similar to node v in terms of structural proximity, no matter whether they are directly linked to node v or not. The structural proximity is measured by a distance function dis(∙, ∙) that is defined in the latent space *ℝ*^d^ as follows:

(3) $$\begin{array}{c} dis\left(z_{v},z_{u}\right)⟶r\in R\text{,} \end{array}$$

where *r* represents the structural proximity between the nodes *v* and *u* in the latent space. Subsequently, we sort the distance *r* from small to large and include the nodes in a certain range of structural proximity into the neighborhood *𝒩*_z_(v). Let [start, en d] denote the range, the structural neighborhood *𝒩*_z_(v) is defined as follows:

(4) $$\begin{array}{c} N_{z}\left(v\right)=\left\{\left.u\right|u\in V,start\leq \#dis\left(z_{v},z_{u}\right)\leq end\right\}, \end{array}$$

where #dis(z_v_, z_u_) means the position of the distance di s(z_v_, z_u_) in the sorted queue of *r*.

The EMPG *𝒢*′=(*𝒱*, *ℰ*′) is constructed according to *𝒩*_z_(v) afterward. If u ∈ *𝒩*_z_(v) and (u, v) ∉ *ℰ*, an edge (u, v) is added to the graph *𝒢*=(*𝒱*, *ℰ*). Therefore, *ℰ*′=(u, v) ⋃ *ℰ*. An example of EMPG is shown in the lower left corner of Figure 1. In the EMPG *𝒢*′=(*𝒱*, *ℰ*′), with the help of the added connections, a node can propagate its message to other nodes that are long distance from it in the original graph but possess a similar structure.

Our approach to determining the structural neighborhood is totally different from the existing work. For example, Kampffmeyer et al. [26] use the path distance between nodes to weight the contribution of different nodes. Pei et al. [28] set a structural proximity threshold to extract the neighborhood first, and then added connections between the nodes in the neighborhood. However, this way of adding connections changes the node degree distribution of the input graph. Additionally, it easily leads to the appearance of large degree nodes. Our way of adding edges does not change the shape of node degree distribution, since the number of edges added to each node is nearly same, that is about (end − start). Furthermore, our way would not generate nodes with much high degree. A node with large degree is more likely to suffer from over-smoothing in a multilayer GCN, since the repeatedly applying Laplacian smoothing will converge to be proportional to the square root of node degree [22, 27].

#### 3.1.3. Message Propagation Enhancement

In a layer of GCN, each node sends its message to its neighbors, and then updates its feature representation by aggregating all messages received from its neighbors. The messages from the neighbors with the same label bring positive influences on node classification, whereas the messages from the neighbors with different label bring negative influences. The added connections should make more nodes receive positive influences more than negative influences from their neighbors. To measure the enhancement of message propagation brought by the added connections, we define a concept named influence range of message propagation, which is a novel metric that measures the effectiveness of a dense connection scheme quantitatively.

Given a node *v*_*i*_ ∈ *𝒱* and a *k*-layer GCN, the node *v*_*i*_ can receive the messages propagating from the nodes at *k*-hop distance in the graph. When the recursive learning process ends, the influence that the node *v*_*i*_ receives from other nodes in the graph can be defined as follows:

(5) $$\begin{array}{c} influence\left(v_{i}\right)={influence}^{p}\left(v_{i}\right)+{influence}^{n}\left(v_{i}\right), \end{array}$$

where influence^*p*^(*v*_*i*_) and influence^*n*^(*v*_*i*_) represent the influence received by *v*_*i*_ from the nodes with the same label and from the nodes with different label, respectively. For a *k*-layer SGC defined by (2), influence^*p*^(*v*_*i*_) and influence^*n*^(*v*_*i*_) are defined, respectively, as follows:

(6) $$\begin{array}{c} {influence}^{p}\left(v_{i}\right)=\underset{j\in V}{\sum }\underset{l\in C}{\sum }{\hat{s}}_{i,j}^{k}∙\delta \left(Y_{i,l}=Y_{j,l}\right),\\ {influence}^{n}\left(v_{i}\right)=\underset{j\in V}{\sum }\underset{l\in C}{\sum }{\hat{s}}_{i,j}^{k}∙\delta \left(Y_{i,l}\neq Y_{j,l}\right), \end{array}$$

where *δ*(*∗*)=1 if the condition *∗* is satisfied; otherwise, *δ*(*∗*)=0.

The influence range of message propagation is defined as the ratio of the number of nodes that receive positive influences more than negative influences to the total of nodes. That is,

(7) $$\begin{array}{c} influence\;range=\frac{\sum_{v_{i}\in V}\delta \left(influence\left(v_{i}\right)>0\right)}{\left|V\right|}. \end{array}$$

As an example, Figure 3 shows the positive influence (blue) and the negative influence (orange) received by each node in message propagation in the original Cora [51] network (upper) and the enhanced Cora network (lower), respectively. The red points on the horizontal axis mean the corresponding nodes are labeled nodes. Because of edge sparsity and label scarcity, some nodes in the original graph cannot receive messages from the labeled nodes or receive negative messages only. The influence range of message propagation increases from 33.35% in the original graph to 59.23% in the enhanced graph.

Besides measuring the improvement of message propagation, the concept of influence range of message propagation can also be used to indicate message propagation saturation. When the influence range of message propagation no longer increases, the message propagation reaches saturation.

### 3.2. Constructing Multi-Channel GCNs on Dropout EMPGs

With the aid of the added connections, a node's message can propagate to the nodes at long distances, without the need of increasing convolutional layers. However, the added connections may bring noise. Additionally, too dense connections are more likely to cause message propagation saturation. What is worse, the GCN constructed on the EMPG directly is prone to overfit the few training data, since each layer has numerous trainable parameters. A reasonable understanding of the EMPG is to regard it as an accumulation of some potential variants of the original graph. In this step, dropout is used to extract reasonable variants from the EMPG first. Subsequently, the multi-channel GCNs are built on the different variants, whose outputs are aggregated to produce the final representation.

Dropout was first introduced by Hinton et al. [41] as a way to train deep neural networks, in which a collection of hidden neurons is stochastically “dropped out” at each iteration of a training procedure. It has been proven effective in controlling overfitting. Dropout can be understood as a regularizer. Alternatively, dropout can be seen as averaging over many neural networks with shared weights [52]. Dropout also reduces model complexity and therefore improves computational efficiency [53]. Here, we use dropout as a data augmentation technique. A group of variants of the input graph is generated by repeatedly removing edges from the EMPG randomly, each of which is used as a substitute for the input graph to train the GCNs on different channels.

We apply dropout to the edges of the EMPG *𝒢*′=(*𝒱*, *ℰ*′). Each edge (v_i_, v_j_) ∈ *ℰ*′ is removed with a probability *p*, independent of others. A dropout EMPG is denoted by *𝒢*′=(*𝒱*, *ℰ*_drop_′), whose adjacency matrix A_drop_′ is calculated by A_drop_′=R*∗*A′. R ∈ {0, 1}^|*𝒱*|×|*𝒱*|^ is a random matrix that is generated according to the generative process r_i,j_ ~ Bernoulli(1 − p). A′ is the adjacency matrix of the EMPG *𝒢*′=(*𝒱*, *ℰ*′) and the symbol ∗ means an element-wise product. As shown in Figure 1, the GCNs are constructed on various dropout EMPG *𝒢*′=(*𝒱*, *ℰ*_drop_′). For the *i*-th channel, the re-normalization trick is performed on A_i−drop_′, leading to ${\hat{A}}_{i-drop}^{\prime }={\hat{D}}^{-1/2}\left(A_{i-drop}^{\prime }+I\right){\hat{D}}^{-1/2}$. The feed-forward propagation in the *i*-th channel GCN is recursively conducted as follows:

(8) $$\begin{array}{c} H_{i}^{\left(k+1\right)}=ReLU\left({\hat{A}}_{i-drop}^{\prime }H_{i}^{\left(k\right)}W_{i}^{\left(k\right)}\right)\text{.} \end{array}$$

The last but not least step is to aggregate the features H_i_^(k)^obtained from different channels to compute the final prediction. Because it is reasonable to regard the features learned from different dropout EMPGs as equally important, we aggregate the features H_i_^(k)^ just by summarizing them together as:

(9) $$\begin{array}{c} H^{\left(k\right)}=\underset{i}{\sum }H_{i}^{\left(k\right)}\text{.} \end{array}$$

The process of constructing multi-channel GCNs described above is different from the existing work. For example, Rong et al. [43] adopted the technique of dropping edges also. The major difference between their method and ours is that our method applies dropout to the EMPG, whereas their method applies dropout to the input graph directly, which is certainly not workable when the input graph is sparse. In order to boost GCN robustness, Ioannidis and Giannakis [54] added and removed edges with probabilities to simulated noise. In contrast, we use dropout to augment training graphs and increase robustness by combining multi-channel outputs. More importantly, our way of generating training graphs by dropping EMPG edges can make the augmented training graphs possess the same underlying distribution of the input graph. Preserving the distribution of training data has been proved to be critical to training classifiers [55]. Because the training graphs in different channels have the same distribution, we can aggregate the multi-channel features directly by summation without loss of accuracy. In contrast, to guarantee classification accuracy, Peng et al. [56] measured the weight of the feature map of each channel of each subgraph by a self-attention mechanism while concatenating them into a vector. The two seemingly contradictory steps in our method, adding links elaborately and removing edges randomly, actually complement one another and make a difference in the task of node classification in sparse graph with few labels.

### 3.3. Complexity Analysis

Now we analyze the computational complexity of the proposed method. We use aggregate analysis, which counts up the complexity of each step and uses the sum to determine the total complexity. As described in Section 3.1, the first step of the proposed method is to embed each node of the input graph *𝒢*=(*𝒱*, *ℰ*) to a vector space *ℝ*^d^ through DeepWalk [48]. As we know, DeepWalk first generates *γ* random walks of fixed length q from each node, and then utilizes the skip-gram model, which maximizes the cooccurrence probability among the nodes that appear within a *ω*-width window in a random walk, to embed the input graph. The time complexity of DeepWalk is Ο(*γ*|*𝒱*|q*ω*(d+dlog|*𝒱*|)) [57]. As the parameters *γ*, q, *ω*, and d are small integers, we can say DeepWalk runs in a time bounded by Ο(|*𝒱*|log|*𝒱*|) for the sake of simplicity.

After embedding the input graph, the proposed method generates the EMPG *𝒢*′=(*𝒱*, *ℰ*′) using formula (3) and (4). The time complexity of generating EMPG is bounded by Ο(|*𝒱*|^2^), because the distance between all pairs of nodes in the latent space *ℝ*^d^should be calculated. While constructing *𝒩*_z_(v), we use a randomized-select algorithm that returns the i-th smallest distance on average in linear time.

The next step of the proposed method is to generate the dropout EMPG *𝒢*′=(*𝒱*, *ℰ*_drop_′) from the EMPG *𝒢*′=(*𝒱*, *ℰ*′). The time complexity of this step is Ο(|*𝒱*|^2^) because of the element-wise product A_drop_′=R*∗*A′.

The last step is to build a GCN on each dropout EMPG *𝒢*′=(*𝒱*, *ℰ*_drop_′) for every channel. Because the GCN in each channel can be trained independently, we analyze the complexity of a channel only. We build a two-layer SGC in each channel. The complexity of a two-layer SGC is Ο(2|*ℰ*_drop_′|d) [58]. Because |*ℰ*_drop_′| ≈ |*ℰ*|, the complexity of this step is Ο(2|*ℰ*|d). Thus, the overall time complexity is Ο(|*𝒱*|log|*𝒱*|)+Ο(|*𝒱*|^2^)+Ο(|*𝒱*|^2^)+Ο(2|*ℰ*|d) = Ο(|*𝒱*|^2^). It is worth to note that the re-normalization of each adjacency matrix A_drop_′ can be computed in advance and each dropout EMPG *𝒢*′=(*𝒱*, *ℰ*_drop_′) is sparse, i.e., |*ℰ*_drop_′| ≪ |*𝒱*|^2^. Thus, the execution time can be reduced significantly by using parallel calculation.

## 4. Experiment and Discussion

The effectiveness of the proposed method was evaluated on the task of semi-supervised node classification in two citation networks, Cora [51] and Citeseer [59]. In this section, the experimental results are presented and comprehensively analyzed to illustrate the key properties of the proposed method.

### 4.1. Datasets and Experimental Setup

The experiments were conducted on two real-world citation datasets: Cora and Citeseer. Their statistics are reported in Table 1. Please note that the edge density of Citeseer is much lower than that of Cora. The edge density influences method performance. The experimental results described below indicate that the scheme of enhancing message propagation is more effective for sparse graphs.

Each dataset was split into three parts in the experiments: 1%–5% labeled data in each class were randomly selected for training, 500 for validation, and 1000 for the test. A two-layer SGC was built by using PyTorch and trained for 600 epochs by using Adam with learning rate 2e-2. The L2 regularization parameter was set to 5e-4. In addition, step decay schedule was used to drop the learning rate by 0.97 half every 60 epochs. The experiments that investigated the influence of a certain factor on the method performance used the same parameter settings. However, delicate parameter selection was performed in the experiments of pushing node classification accuracy.

All experiments run on a machine with an Intel (R) Core (TM) i7-10700 CPU 2.90 GHz with 16 threads and 256 GB memory. We first generated 10 dropout EMPGs from the input graph and then trained the two-layer SGC of each channel one by one. The time spent on generating the dropout EMPG from Cora and Citeseer is about 80.6 and 104.7 seconds, respectively. The execution time for training a two-layer SGC in a channel for Cora and Citeseer is 0.41 and 0.57 seconds, respectively. The time spent on preparing the training graphs of the multi-channel SGCs dominates the overall running time. However, because the multiple channels are independent of each other, the time cost can be controlled at low level by using parallel calculation.

The classification accuracy was used as a metric to evaluate the performance of the proposed method on the task of semi-supervised node classification, which is defined as follows:

(10) $$\begin{array}{c} Accuracy=\frac{n_{correct}}{n_{total}}\text{.} \end{array}$$

It is the ratio of the number of correct classifications *n*_correct_ to the total number of test data *n*_total_.

### 4.2. Experimental Results

#### 4.2.1. Enhancement of Influence Range

The aim of adding connections is to enlarge the influence range of message propagation, since a small influence range cannot lead to a high accuracy of node classification.  Figure 4 compares the influence range of message propagation in the original graph (blue) and the enhanced graph (orange) with the increasing label rate on Cora (upper) and Citeseer (lower) datasets, respectively. It can be observed from the left of Figure 4 that the influence range of message propagation in the enhanced graph is always larger than that in the original graph. This is as expected, because the added connections provide more paths for message propagation. When only few labeled nodes are given (<3%), the added connections lead to a rapid increase in the influence range. When the label rate continuously rises above 10%, the influence range of messages propagation nearly covers the entire graph, that is, nearly reaches saturation. The green curves on the right of Figure 4 show the enhancement of influence range, which increases fast initially and drops gradually when the training label rate increases over 3%. In addition, with the same training label rate, the enhancement of influence range in Citeseer is larger than that in Cora. The reason is that the edge density of Citeseer is much lower than that of Cora. The added connections play a relatively much more important role in message propagation in Citeseer than in Cora.

#### 4.2.2. Accuracy of Node Classification

This experiment reveals how the accuracy of node classification benefits from the enhancement of influence range.  Figure 5 shows the accuracy of node classification in the original graph (blue) and the enhanced graph (orange) as the training label rate increases from 1% to 20% on Cora (upper) and Citeseer (lower) datasets. For Cora, the accuracy obtained on the enhanced graph is consistently better than that obtained on the original graph. For Citeseer, when very few labeled nodes are given for training (<3%), the improvement on classification accuracy is evident. When the label rate increases from 3% to 10%, the classification accuracy obtained on the enhanced graph is still better but the gap drops. When the label rate increases over 10%, the improvement is very limited and sometimes the accuracy may get worse. The green curves on the right of Figure 5 show the improvement on classification accuracy. Compared with the enhancement of influence range shown on the right of Figure 4, the tendency of the improvement of classification accuracy is consistent with the tendency of the enhancement of influence range for both datasets, which means the influence range of message propagation is critical to node classification accuracy and enlarging influence range via adding connections really improves node classification accuracy. However, when the training label rate is larger than 10%, the influence range of message propagation is close to saturation. As a result, the classification accuracy either increases a little bit or even decreases.

Table 2 compares the node classification accuracy of our method with that of seven baseline methods on Cora and Citeseer datasets. The reported numbers in Table 2 denote the node classification accuracy in percent. The results of the benchmark methods were taken from the relative references. All experiments were run on the same fixed split of 5% labeled nodes of each class for training, 500 nodes for validation, 1,000 nodes for test, and the rest of nodes as unlabeled data, which is the standard split used in most method evaluations [49].

The last column of Table 2 lists the node classification accuracies of all methods on the Citeseer dataset. Our method significantly outperforms all the seven competing methods on the Citeseer dataset. This clearly indicates the performance advantage of our method over the existing methods for node classification in graphs that are very sparse and have few labeled nodes, like the citation network Citeseer. The reason is that the added connections play a relatively much more important role in message propagation in very sparse graphs.

The middle column of Table 2 lists the node classification accuracies of all methods on the Cora dataset. Our method outperforms six of the seven competing methods and achieves an accuracy as equally good as DGCN [12]. DGCN combines two-channel GCNs, one learns the local consistency from the adjacency matrix and another learns global consistency from Positive Pointwise Mutual Information (PPMI) matrix. In contrast, our method adopts multi-channel GCNs to aggregate the features learned from different dropout EMPGs. Both methods emphasize the importance of performing graph convolution from different views of the input graph. That may be the reason why both methods outperform other six methods on the two benchmark datasets and perform equally well on the Cora dataset. However, DGCN employs random walks to build the PPMI matrix. Compared to the Cora network, the Citeseer network is much sparser, where most nodes are separated from each other. It is difficult for random walk to collect the global structural information of a very sparse graph, because random walk cannot reach the separated nodes. Whereas our method utilizes random walk to collect local structural information around each node when embedding the original graph, but exploits the information of long-range nodes through the added connections. That may be the reason why our method outperforms DGCN on the Citeseer dataset.

Furthermore, we compare the computational complexity of DGCN with that of our method. The time complexity of generating the PPMI matrix is Ο(*γ*|*𝒱*|q^2^)+Ο(|*𝒱*|^2^), the former is the complexity of random walks and the latter is the complexity of constructing the PPMI matrix. DGCN uses a dual graph convolutional architecture with two graph convolutional layers in each channel, whose complexity is Ο(2(|*𝒱*|^2^d+|*𝒱*|d^2^)). Therefore, the complexity of DGCN is also bounded by Ο(|*𝒱*|^2^). However, because the PPMI matrix is not sparse, the upper bound Ο(|*𝒱*|^2^) of DGCN cannot be reduced to Ο(|*ℰ*|), like in the case of sparse dropout EMPG. Additionally, DGCN uses two-layer GCNs and Batch Gradient Decent (BGD) to train the GCNs in order to achieve good accuracy, whereas our method uses two-layer SGCs and Stochastic Gradient Decent (SGD) to train the SGCs. SGC runs faster than GCN and BGD is slower than SGD. Therefore, DGCN is relatively slow in practical calculation, which was also pointed out by the authors of [12]. Our method achieves classification accuracy equal to or better than that DGCN yields without loss of efficiency.

Additionally, it is worth noting that our model outperforms the original SGC [8] by obvious margins on both benchmark datasets. Our method constructs a two-layer SGC in each channel to learn feature representations from different dropout EMPGs and then combines the multi-channel outputs together. However, SGC [8] learns feature representation directly from the original graph. The accuracy improvement proves that the scheme of adding connections and the strategy of augmenting training samples by dropout are indeed helpful for improving node classification accuracy. It is convenient to incorporate other GCNs into the framework shown in Figure 1. It is rational to expect that the proposed method may yield better classification accuracy when incorporating other appropriate GCNs.

#### 4.2.3. Effect of Densification Strength

The pair of parameters [start, end] affect the accuracy of node classification. The value (end − start) indicates how many connections are added to each node of the original graph, which represents the densification strength.  Figure 6 shows the accuracy of node classification on Cora (left) and Citeseer (right) datasets when the parameters start and en d change from 0 to 9, given three different training label rates 1% (up), 2% (middle), and 5% (down). The block color represents the value of accuracy, with lighter colors indicating higher values and darker colors indicating lower ones. It can be found that our method achieves good classification accuracy when the parameter start is set a little less than the average node degree and the parameter en d is set around double the average node degree. This is understandable, as there is a high probability that the nodes with the closest proximity have already been connected directly in the original graph. On the other hand, setting a smaller start or/and a larger en d to add more than double edges will not only bring more noise but also make message propagation saturate soon.

#### 4.2.4. Effect of Dropout Rate

The dropout rate p is a tunable parameter that indicates the probability of removing the edges of the EMPG *𝒢*′=(*𝒱*, *ℰ*′). We increased it from 0 to 0.9 with an increment of 0.1 to examine how the classification accuracy depends on it. Meanwhile, the densification strength [start, en d] was set from the average node degree to double the average node degree.  Figure 7 shows the validation accuracy (blue) and the test accuracy (yellow) for varying dropout rate p on Cora (left) and Citeseer (right) datasets with the training label rate 1% (up), 2% (middle), and 5% (down). A large p means few edges of the EMPG *𝒢*′=(*𝒱*, *ℰ*′) are retained for message propagation. For the training label rate 1% and 2%, both the validation accuracy and the test accuracy on Cora continue to increase till p reaches 0.8, followed by a rapid drop. However, for the training label rate 5%, both accuracies increase till a larger value of p. The curves on the right of Figure 7 show that the validation accuracy and the test accuracy on Citeseer drop continuously with the increasing dropout rate p for the training label rate 1% and 2%. For the training label rate 5%, the validation accuracy and the test accuracy on Citeseer increase till p=0.4 and then take a turn for the worse.

The clue to the complex trends of both accuracies appears when considering the average edge density, the densification strength (end − start), the dropout rate p, and the training label rate jointly. The influence range of message propagation is determined by all these factors that work together. No matter which factor changes, if it expands the influence range, the accuracy will increase. Otherwise, the accuracy will decrease. Adding connections enhances message propagation but dense connections may lead to message propagation saturation as the label rate increases. On the other hand, removing edges reduces noise and prevents message propagation saturation. Generating various dropout EMPGs can be viewed as a way of augmenting training data. Using a group of complementary data to train model jointly is helpful for mitigating overfitting. The two seemingly contradictory operations, adding connections deliberately and removing edges randomly, play different roles, which actually complement one another and work together to improve the accuracy of node classification.

#### 4.2.5. Analysis of Robustness

Robustness is important for a GCN to obtain high accuracy when graph data contain noise. To study the influence of different noise levels on the accuracy of node classification, we randomly selected 10% to 50% samples from the training dataset, changed their labels, and then used the changed training dataset to train the model.  Figure 8 depicts the accuracy obtained in the original graph (yellow) and the enhanced graph (blue) for varying noise level on Cora (left) and Citeseer (right), given three different training label rates of 1% (up), 2% (middle), and 5% (down). It is clear that the accuracy decreases as the noise level increases. However, for Cora, the accuracy obtained on the EMPG is consistently better, and the gap is obvious and enlarges as the noise level increases. For Citeseer, with the low training label rate of 1% and 2%, the accuracy obtained on the EMPG fluctuates up and down around the accuracy obtained on the original graph. When the training label rate increases to 5%, the accuracy obtained on the EMPG is always better than the accuracy obtained on the original graph, but the gap decreases as the noise level increases. To sum up, the model built on the enhanced graph is more robust than the model built on the original graph.

## 5. Related Work

In the past few years, a number of methods for improving message propagation in GCNs have been proposed, most of which fall into two broad categories: the methods toward building deep GCN and the methods based on dense connection scheme. This section presents an overview of the related work in both fields.

### 5.1. Methods Toward Building Deep GCN

A straightforward solution to realize long-range message propagation is to deepen GCN. However, a serious problem in deep GCNs is over-smoothing, which was first discussed in [22]. To exploit the strengths and overcome weaknesses of deep GCN, Xu et al. [24] proposed JK-network, which enables different neighborhood ranges and employs skip connections to realize multi-hop message propagation. Li et al., [25] used residual connections and dilated convolutions to facilitate the building of deep GCN. GCNII, a simple and deep network that prevents over-smoothing by residual connections and identity mapping, was proposed in [27]. Sun et al. [47] proposed an RNN-like deep network called AdaGCNs, which uses AdaBoost to combine the predictions from different order neighbors when building deep network, rather than only stacking a specific type of graph convolutional layer. Zhang et al. [60] built a residual dense deep network that extracts local features via densely connected convolutional layers. Klicpera et al. [61] proposed a message propagation scheme based on personalized Pagerank, by which they successfully built a deep network that can use the message from a large and adjustable neighborhood. DAGNN [62] incorporates the information from large receptive fields through the entanglement of representation transformation and propagation. Zhao et al. [63] added a normalization layer into graph neural network architecture, by which they could stack more layers into a network. Wenkel et al. [64] proposed a hybrid deep GNN framework that combines traditional GCN filters with band-pass filters to combat over-smoothing. These efforts have produced promising results. However, stacking a large number of convolutional layers leads to more complex models with more parameters. Training such complex models is challenging especially in semi-supervised classification. And what is worse, the deep networks with too many trainable parameters are very prone to overfitting when the labeled data are scarce.

### 5.2. Methods Based on Dense Connection Scheme

On the other hand, some researchers attempted to improve message propagation with shallow neural networks. For example, SGC [8] uses the *k*-th power of graph convolution matrix in a layer to capture higher-order information. GAT [9] learns the weight of messages from different neighbors and improves message aggregation by an attention mechanism. Thekumparampil et al. [10] removed all the intermediate fully connected layers and replaced the propagation layers with an attention mechanism to improve message aggregation. A dual graph convolutional network that considers local and global information together was proposed in [12] to deal with semi-supervised node classification. Xu et al. [13] proposed GIL that uses between-node paths to propagate messages between long-range nodes. Kampffmeyer et al. [26] proposed DGP that uses a weighted dense connection scheme to select links among distant nodes to improve message propagation. To extract long-range structural information for aggregation, Pei et al. [28] rebuilt the structural neighborhood by adding connections into the input graph according to graph embedding. The major difference between their work and ours lies in the way of selecting neighbors and utilizing the added connections. Our method employs dropout to avoid the side effects of dense connections and adopts a multi-channel aggregation architecture. Whereas the method proposed in [28] uses a bi-level aggregation scheme to update node features and combats computational complexity by controlling the number of virtual nodes. The shallow models with dense connection scheme are more effective than the shallow models without enhanced message propagation scheme. Compared to deep networks, shallow models are usually computationally efficient because the number of layers is small.

Our method belongs to the second category. The major difference compared with these works mentioned above lies in the way of adding and using dense connections. Our method adds connections according to graph embedding and keeps the shape of node degree distribution unchanged after adding connections. Furthermore, our method constructs multi-channel GCNs on different dropout EMPGs to extract features from different views for aggregation, which can leverage the strengths of the added connections and avoid their negative impacts simultaneously.

## 6. Conclusion and Future Work

In this article, a new GCN framework is proposed to address the problem of semi-supervised node classification in sparse graph with few labels, whose distinguishing feature is a dense connection scheme based on graph embedding, by which the GCN can collect the messages from the right nodes at long distances efficiently. Thus, the proposed method need not stack multiple convolutional layers into a GCN, which is very useful for avoiding over-smoothing and reducing model complexity. Meanwhile, the multi-channel GCN architecture mitigates the negative effects of dense connections and prevents overfitting by learning with augmented data, which finally improves the accuracy of node classification. The experiments on benchmark datasets demonstrate the effectiveness of the proposed method for solving the problem of node classification in sparse graph with few labeled nodes. Furthermore, the proposed method is robust and efficient.

In future work, we plan to explore mechanisms for adding connections adaptively and dynamically. It will be worthwhile to model the relationship among graph properties, edge densification strength, and message propagation range, which would be useful for preventing message propagation saturation. We will also apply the proposed method to solve more real-world problems.

## Figures and Tables

**Figure 1:** The framework of the proposed method.

**Figure 2:** The organization of GCN and the recursive training process.

**Figure 3:** The positive influence (blue) and the negative influence (orange) received by each node in message propagation in the original Cora network (a) and the enhanced Cora network (b).

**Figure 4:** Comparisons of the influence range in the original graph (blue) and the enhanced graph (orange) as the training label rate increases on Cora (a) and Citeseer (b) datasets.

**Figure 5:** Accuracy obtained in the original graph (blue) and the enhanced graph (orange) as the training label rate increases on Cora (a) and Citeseer (b) datasets.

**Figure 6:** Accuracy for varying start and end on Cora (left) and Citeseer (right) datasets with training label rate 1% (a), 2% (b), and 5% (c).

**Figure 7:** Validation accuracy (blue) and test accuracy (yellow) for varying dropout rate *p* on Cora (left) and Citeseer (right) datasets with training label rate 1% (a), 2% (b), and 5% (c).

**Figure 8:** Accuracy obtained in the original graph (yellow) and the enhanced graph (blue) for varying noise level on Cora (left) and Citeseer (right) datasets with training label rate 1% (a), 2% (b), and 5% (c).

**Table 1:** Dataset statistics.

Dataset	Nodes	Edges	Classes	Features	E-Den (%)	N-Deg
Cora	2708	5429	7	1433	0.148	4.01
Citeseer	3327	4732	6	3703	0.086	2.84

**Table 2:** Summary of node classification accuracy.

Model	Cora	Citeseer
DeepWalk [48]	67.2	43.2
GCN [7]	81.5	70.3
SGC [8]	81.0	71.9
GAT [9]	83.0	72.5
AGNN [10]	83.1	71.7
TAGCN [11]	83.3	71.4
DGCN [12]	83.5	72.6
Our method	83.5	73.3

## Data Availability

The two public datasets used in this article, Cora and Citeseer, can be downloaded from https://linqs-data.soe.ucsc.edu/public/lbc/cora.tgz and https://linqs-data.soe.ucsc.edu/public/lbc/citeseer.tgz, respectively.
